The article "Eight-Year Trend Analysis of Cutaneous Leishmaniasis Cases in West Amhara Region Referred to Amhara Public Health Institute Northwest, Ethiopia: A Retrospective Study" was published in 2022. Journal: Biomed Res Int.

# Eight-Year Trend Analysis of Cutaneous Leishmaniasis Cases in West Amhara Region Referred to Amhara Public Health Institute Northwest, Ethiopia: A Retrospective Study

**DOI:** 10.1155/2022/6562092

**Published:** 2022-08-22

**Authors:** Banchamlak Tegegne, Mulat Yimer, Kefale Ejigu, Getaneh Alemu, Fikirte Estifanos

**Affiliations:** ^1^Amhara Public Health Institute, Bahir Dar, Ethiopia; ^2^Department of Medical Laboratory Sciences, School of Health Sciences, College of Medicine and Health Sciences, Bahir Dar University, Bahir Dar, Ethiopia

## Abstract

Cutaneous leishmaniasis is a continually spreading health problem in Amhara Region, Ethiopia. Despite this, up- to-date information on referral laboratory facility has been not yet reported. Therefore, this study was aimed at reporting up-to-date information about eight year's cutaneous leishmaniasis trend status. Data on referred cases from 2013 to 2020 were collected at Amhara Public Health Institute Parasitology department by reviewing log book. Of the 243 suspected cases, 114 (46.9%) were positive (confirmed) with microscope and cultured results showed that most of them were negatives. Most of the suspected cases were from 16 to 30 years and males by age and sex, respectively. Trend status by year depicted that largest numbers of suspected and confirmed cases were reported in 2013, 2015, and 2019 years. Finally, the trend status by zone showed that most cases were reported from South Gondar and Awi zones, respectively.

## 1. Introduction

Leishmaniasis is epidemiologically and clinically diverse disease caused by protozoan parasites of the genus *Leishmania* [1]. It is transmitted by the bite of the female *Phlebotomus* species in the Old World and *Lutzomyia* species in the New World [1, 2]. The clinical outcome of the disease might vary depending on the infecting *Leishmania* species and/or the immune status of the host and some other factors. Hence, some species infect the visceral organs while others are dermotrophic and infect the skin [3]. As a result, clinical manifestations of leishmaniasis can be grouped into two as follows: cisceral leishmaniasis (VL), caused by *L*. *donovani* complex (*L*. *donovani* and/or *L*. *infantum*) and cutaneous leishmaniasis (CL), caused by *L*. *major*, *L*. *tropica*, *L*. *aethiopica*, *L*. *braziliensis*, and *L*. *mexicana* species complex [4–6].

Recent reports in 2022 depicted that over 85% of new CL cases occurred in 10 countries: Afghanistan, Algeria, Brazil, Colombia, Iraq, Libya, Pakistan, Peru, the Syrian Arab Republic, and Tunisia. It is estimated that between 600 000 and 1 million new cases occur worldwide annually. Despite this, over 90% of mucocutaneous leishmaniasis cases occur in Bolivia, Brazil, Ethiopia, and Peru [7].

The article "Eight-Year Trend Analysis of Cutaneous Leishmaniasis Cases in West Amhara Region Referred to Amhara Public Health Institute Northwest, Ethiopia: A Retrospective Study" was published in 2022. Journal: Biomed Res Int.

Cutaneous leishmaniasis is a growing health problem in Ethiopia [8], and currently, it is endemic in 80 districts with 20,000 to 30,000 incidence cases and 29 million people are at risk of infection [9]. It is caused by *L*. *aethiopica* transmitted by bite of *Phlebotomus longipes* and *Phlebotomus pediffer* in the highland areas [10] and rarely, *L*. *tropica* and *L*. *major* transmitted by bite of *Phlebotomus sergenti* and *Phlebotmus duboscqi* in the low land areas, respectively [10, 11]. It presents in three clinical forms: localized cutaneous leishmaniasis (LCL), mucocutaneous leishmaniasis (MCL), and diffused cutaneous leishmaniasis (DCL) [6, 12].

Even if the disease has significant social and medical impacts, the attention given to prevention and control has been comparatively poor [13]. As a result, nowadays, CL is spreading to the new foci and there is also occurrence of outbreaks in Siltie district southern Ethiopia [14]. Outbreaks had also been occurred with undulating pattern at Dega Damot and Ankesha-Guagusa districts in the Amhara Region [15, 16]. Despite this problem, a few data were reported on peripheral health facilities. However, up-to-date information on referral laboratory level has been not yet reported. Moreover, this study will have an input for the control program by the government. Therefore, this study is aimed at assessing the eight-year retrospective study of CL cases referred to Amhara Public Health Institute northwest, Ethiopia.

## 2. Materials and Methods

### 2.1. Study Design, Area, and Period

The eight-year retrospective study was conducted by reviewing laboratory registration books from CL suspected cases recorded at Amhara Public Health Institute (APHI) from December 2020 to January 2021. Previously, the institute was named as the Amhara regional laboratory and stablished in 1996 and had been worked as a reference laboratory by confirming different laboratory tests that were not done at peripheral hospitals level. Later, it was grown to APHI in 2015 and serve as a technical arm of the Amhara Regional Health Bureau, and since then, it has served as a research center for the region and acts as a center for laboratory confirmation of different tests that have been referred from peripheral heath facilities in the Amhara region. The headquarter of the institute has been situated in Bahir Dar City, Ethiopia. This headquarter institute has branched institutes at Dessie, Woldyia, Debre-Markos, and Debre-Tabor towns. In addition, the branched institutes support the nearby health facilities as a reference laboratories and the headquarter institute also supports nearby health facilities. Moreover, the head quarter also composed of three main directorates: public health emergency management, research development, and laboratory directorates. The laboratory directorate has seven reference laboratories of which parasitology reference laboratory is one of them. This reference laboratory is internationally accredited by ISO15189 standard on *Leishmania* microscopy and *Leishmania* culture since 2018.

The article "Eight-Year Trend Analysis of Cutaneous Leishmaniasis Cases in West Amhara Region Referred to Amhara Public Health Institute Northwest, Ethiopia: A Retrospective Study" was published in 2022. Journal: Biomed Res Int.

### 2.2. Data Collection

Cutaneous leishmaniasis suspected cases are referred to APHI for diagnosis of CL whenever one or two or all the following conditions had occurred: (1) if there is no laboratory facility or logistics at peripheral health facilities, (2) if the clinical manifestations are suggestive of CL but skin slit microscopy revealed negative result, and (3) if a patient is nonresponsive to drugs or if repeated relapse occurs. When suspected cases are referred to APHI Parasitology reference laboratory for CL diagnosis, both skin slit microscopy and culture using Novy-MacNeal-Nicolle (NNN) media have been performed by trained and well experienced parasitologists. Accordingly, results of both the smear microscopy and culture are reported. Skin slit sampling for culture needs to be sterile, and usually, it is difficult to do so and liable for contamination and mostly cultures contaminated in the early period of incubation (from seven to eight days post inoculation). As a result, culture from significant number of samples became unreliable result. Moreover, previously, there were interruption of culture service due to laboratory logistics supply. In such cases, results are reported merely on skin slit microscopy.

Information on sociodemographic characteristics, clinical data of CL suspected cases and skin slit microscopy, and culture results were collected from the patient log book using Excel sheet version 10. Accordingly, suspected cases diagnosed in the institute from 2013 to 2020 were included in the study since regular referral system was started in 2013. Patients referred for laboratory diagnosis for one of the three clinical forms of CL and came from West Amhara Zones with age, sex, residence at zonal, and district level, suspected clinical form of CL, and had culture, and/or microscopy results were included in this study.

### 2.3. Skin Slit Sample Processing and Laboratory Examination at APHI

As soon as the referred suspected cases arrived with the request paper at the institute, important patient information were fulfilled in the Laboratory information system (LIS). Then, after cleaning the lesion, using 70% alcohol, skin slit samples were taken from the periphery and inoculated in NNN media near the light flame and incubated at 25-27°C for four weeks. In the meantime, additional skin slit was taken and smeared on a new frosted microscope slide. Smears were air dried, fixed, with absolute methanol and stained with 1 : 10 diluted of Giemsa solution for 10 minutes. After washing off the stain and air-drying steps, slides were examined under the microscope using 100x objective. Positive results were graded according to the Ethiopian ministry of health leishmaniasis diagnosis and treatment guideline [17]. Accordingly, results of culture were reported after four weeks of incubation by inspecting every week. The result was taken as positive if there is growth of motile promastigotes seen under inverted microscope. If there were no growth, the result was taken as negative with in the specified period. Finally, if there was growth of fungal elements within six to seven days post incubation, it was reported as early contamination.

The article "Eight-Year Trend Analysis of Cutaneous Leishmaniasis Cases in West Amhara Region Referred to Amhara Public Health Institute Northwest, Ethiopia: A Retrospective Study" was published in 2022. Journal: Biomed Res Int.

### 2.4. Ethical Consideration

Written permission letter was obtained from the APHI research and technology transfer directorate office, and all the information about the patients is remained confidential and used for this study only.

### 2.5. Statistical Analysis

Data collected in Excel sheet were exported to SPSS version 23 for analysis. Descriptive statistics such as line graphs used to present trends by years, zones, and positive (confirmed) cases. Tables were used to present clinical forms of CL by age and sex and laboratory data. During analysis, if a patient record had showed positive result(s) by either skin slit microscopy or culture, it was considered positive.

## 3. Results

Status of CL by age depicted that most (124 (51%)) of the suspected age groups were from 16 to 30 years. Of the three clinical forms, LCL was the most frequently reported type and accounted for 185 (76.1%). On the contrary, the least was DCL and accounted for 6 (13%). Majority 152 (62.6%) of the suspected cases were males (Table 1).

The eight-year trend analysis of CL by year showed that spike in number of suspected and confirmed cases were observed in 2013, 2015, and 2019 years. However, the least numbers of cases were in 2014 and 2016. The trend also depicted that from years 2017 to 2019, there was increment in both suspected and confirmed cases, but in 2018, the number of suspected cases were in decline despite increment in confirmed cases (Figure 1).

Trend status by zone showed that the largest numbers of suspected and confirmed (positive) cases were reported from South Gondar and Awi zones, respectively, while the least numbers of cases were reported from the north Gondar and west Gondar zones. Generally, there were undulating patterns of trends in both suspected and confirmed cases via an eight-year period (Figure 2).

The article "Eight-Year Trend Analysis of Cutaneous Leishmaniasis Cases in West Amhara Region Referred to Amhara Public Health Institute Northwest, Ethiopia: A Retrospective Study" was published in 2022. Journal: Biomed Res Int.

Among the CL suspected cases who were examined using skin slit microscopy, 114 (40.9%) of them were positive (confirmed) cases and most of them had a microscopy result of 1+ followed by 2+. While in culture results, 80 (32.9%) were positive and 10 (4.1%) were early stage contaminations (Table 2).

## 4. Discussion

In this study, status of CL by age depicted that 51% of the suspected age groups were from 16 to 30 years. This was in line with previous studies done at Borumeda Hospital, northeast Ethiopia [18] and at Gondar University Hospital, northwest Ethiopia [19]. But it is was different from studies done at Borumeda Hospital, north east Ethiopia [20] and in Tigray rural communities northern Ethiopia [21]. This difference might be due to difference in age classification in both studies and difference in study setting in the latter case (referral vs. community level).

This study also depicted that LCL was the most frequently reported type and accounted for 76.1% among the three clinical forms and the least reported to be DCL, accounted for 13%. This study was in line with studies done at Gondar University Hospital, northwest Ethiopia [22], at Borumeda Hospital, northeast Ethiopia [20], and in Tigray rural communities, northern Ethiopia [21].

Our study revealed that 62.6% of the suspected cases were males. This study was in line with studies done at Borumeda Hospital, northeast Ethiopia [18, 20], at Gondar University Hospital northwest Ethiopia [19, 21], and in Tigray rural communities northern Ethiopia [22].

## 5. Limitations

Since this is a retrospective study, factors associated with the distribution of CL in the west Amhara region were not addressed. Moreover, molecular tests like PCR was not done to identify the causative species for the three clinical forms of CL.

## 6. Conclusions

Even if, the largest number of suspected and confirmed cases were reported in South Gondar and Awi zones, respectively, our report showed that CL was reported in most of the west Amhara areas. Hence, community awareness and intervention activities should focus on these areas.

## Figures and Tables

**Figure 1:** Trend status of suspected and positive CL cases by year.

**Figure 2:** Trend status of suspected and positive CL cases by zone.

**Table 1:** Clinical forms of cutaneous leishmaniasis by age and sex from 2013 to 2020 in west Amhara region.

		Clinical forms of cutaneous leishmaniasis				
Characteristics		DCL	LCL	MCL	MCL and LCL	Total
		*N* (%)	*N* (%)	*N* (%)	*N* (%)	*N* (%)
Age	<16	0	39 (76.5)	4 (7.8)	8 (15.7)	51 (21)
	16-30	5 (4)	99 (79.8)	15 (12.1)	5 (4)	124 (51)
	31-45	0	19 (86.4)	3 (13.6)	0	22 (9)
	> 45	1 (2.2)	28 (60.9)	11 (23.9)	6 (13)	46 (18.9)
	Total	6 (2.5)	185 (76.1)	33 (13.6)	19 (7.8)	243 (100)
Sex	F	1 (1.1)	75 (82.4)	9 (9.9)	6 (6.6)	91 (37.4)
	M	5 (3.3)	110 (72.4)	24 (15.8)	13 (8.6)	152 (62.6)
	Total	6 (2.5)	185 (76.1)	33 (13.6)	19 (7.8)	243 (100)

The article "Eight-Year Trend Analysis of Cutaneous Leishmaniasis Cases in West Amhara Region Referred to Amhara Public Health Institute Northwest, Ethiopia: A Retrospective Study" was published in 2022. Journal: Biomed Res Int.

**Table 2:** Microscopy and culture results of CL suspected cases referred to APHI from 2013 to 2020 (*n* = 243).

Variable	Category	Frequency, *N* (%)	Total
Smear microscopy	Positive	114 (40.9)	243
	Negative	129 (53.1)	
Grade	1+	42 (36.8)	114
	2+	26 (22.8)	
	3+	19 (16.7)	
	4+	11 (9.6)	
	5+	10 (8.8)	
	6+	6 (5.3)	
Culture results	Positive	80 (32.9)	243
	Negative	100 (41.2)	
	^∗^Early contamination	10 (4.1)	
	Not done	53 (21.8)	

^∗^Early contamination: contamination before 7 days.

## Data Availability

The original data for this study is available from the corresponding author.

## References

[1] Banuls A. L., Hide M., Prugnolle F. (2007). Leishmania and the leishmaniases: a parasite genetic update and advances in taxonomy, epidemiology and pathogenicity in humans. *Advances in Parasitology*.

[2] Cabezas Y., Legentil L., Robert-Gangneux F. (2005). Leishmania cell wall as a potent target for antiparasitic drugs. A focus on the glycoconjugates. *Organic & Biomolecular Chemistry*.

[3] Killick-Kendrick R. (1999). The biology and control of phlebotomine sand flies. *Clinics in Dermatology*.

[4] Scott P., Novais F. O. (2016). Cutaneous leishmaniasis: immune responses in protection and pathogenesis. *Nature Reviews Immunology*.

[5] Kevric I., Cappel M. A., Keeling J. H. (2015). New world and old world leishmania infections: a practical review. *Dermatologic Clinics*.

[6] Savoia D. (2015). Recent updates and perspectives on leishmaniasis. *The Journal of Infection in Developing Countries*.

[7] World Health Organization (WHO) (2020). Global leishmaniasis surveillance, 2017−2018, and first report on five additional indicators. *Weekly Epidemiological Record*.

[8] Gebre-Michael T., Balkewa M., Ali A., Ludovisi A., Gramiccia M. (2004). The isolation of Leishmania tropica and L. aethiopica from Phlebotomus (Paraphlebotomus) species (Diptera: Psychodidae) in the Awash Valley, northeastern Ethiopia. *Transactions of the Royal Society of Tropical Medicine and Hygiene*.

[9] Ethiopian Ministry of Health (2006). Roadmap for neglected tropical diseases operational research in Ethiopia. *NTDs research Advisory Committee (NRAC)*.

[10] Ashford R. W., Bray M. A., Hutchinson M. P., Bray R. S. (1973). The epidemiology of cutane-ous leishmaniasis in Ethiopia. *Transactions of the Royal Society of Tropical Medicine and Hygiene*.

[11] Hailu A., Di Muccio T., Abebe T., Hunegnaw M., Kager P. A., Gramiccia M. (2006). Isolation of Leishmania tropica from an Ethiopian cutaneous leishmaniasis patient. *Transactions of the Royal Society of Tropical Medicine and Hygiene*.

The article "Eight-Year Trend Analysis of Cutaneous Leishmaniasis Cases in West Amhara Region Referred to Amhara Public Health Institute Northwest, Ethiopia: A Retrospective Study" was published in 2022. Journal: Biomed Res Int.

[12] Negera E., Gadisa E., Yamuah L. (2008). Outbreak of cutaneous leishmaniasis in Silti woreda, Ethiopia: risk factor assessment and causative agent identification. *Transactions of the Royal Society of Tropical Medicine and Hygiene*.

[13] Reithinger R., Dujardin J. C., Louzir H., Pirmez C., Alexander B., Brooker S. (2007). Cutaneous leishmaniasis. *Lancet Infect*.

[14] Blum J., Desjeux P., Schwartz E., Beck B., Hartz Z. (2004). Treatment of cutaneous leishmaniasis among travellers. *The Journal of Antimicrobial Chemotherapy*.

[15] Beyene B., Yalew G., Abie G., Abebaw D., Gessese K., Yimer M. An investigation of leshimaniasis outbreak in Dega Damot district, Amhara region, Ethiopia. https://www.researchgate.net/publication/287748430.

[16] Banchamlak T., Mekonnen Y., Tsehaynesh G., Alie A., Mulat Y. (2022). Short reports on cutaneous leishmaniasis outbreak investigation in Ankesha-Guagsa district, Amhara region, Northwest Ethiopia. *Tropical Doctor*.

[17] Ethiopian Ministry of Health (2013). *Guideline for the Diagnosis, Treatment, and Prevention of Leishmaniasis in Ethiopia*.

[18] Bisetegn H., Zeleke A. J., Gadisa E. (2020). Clinical, parasitological and molecular profiles of cutaneous leishmaniasis and its associated factors among clinically suspected patients attending Borumeda Hospital, North-East Ethiopia. *PLoS Neglected Tropical Diseases*.

[19] Ayalew J., Adane D., Arega Y., Rezika M., Helina F. (2021). A ten-year trend of cutaneous leishmaniasis at University of Gondar Hospital, Northwest Ethiopia: 2009-2018. *Journal of Parasitology Research*.

[20] Belayneh E., Hassen M. (2020). Cutaneous leishmaniasis in north-central Ethiopia: trend, clinical forms, geographic distribution, and determinants. *Tropical Medicine and Health*.

[21] Yohannes M., Abebe Z., Boelee E. (2019). Prevalence and environmental determinants of cutaneous leishmaniasis in rural communities in Tigray, northern Ethiopia. *PLoS Neglected Tropical Diseases*.

[22] Fikre H., Mohammed R., Atinafu S., van Griensven J., Diro E. (2017). Clinical features and treatment response of cutaneous leishmaniasis in North-West Ethiopia. *Tropical Medicine & International Health*.

